The article "Application of Multimodal Magnetic Resonance Imaging in Green Channel of Acute and Hyperacute Ischemic Stroke" was published in 2022. Journal: Contrast Media Mol Imaging.

# Application of Multimodal Magnetic Resonance Imaging in Green Channel of Acute and Hyperacute Ischemic Stroke

**DOI:** 10.1155/2022/2452282

**Published:** 2022-07-22

**Authors:** Jianguo Zhou, Guifen Li, Yun Meng, Dayong Fu, Mingcong Lu, Zhi Tang

**Affiliations:** ^1^Department of Radiology, Lianyungang Hospital of Traditional Chinese Medicine, Lianyungang 222004, China; ^2^Department of Radiology, The Second People's Hospital of Lianyungang, Lianyungang 222006, China; ^3^Department of Radiology, The First People's Hospital of Guannan County, Lianyungang 222500, China

## Abstract

The purpose of this study was to observe the effects of multimodal magnetic resonance imaging (MRI) in the green channel of acute and hyperacute ischemic strokes, in order to better guide clinical treatment. The clinical data of 126 patients with acute and hyperacute ischemic stroke who received interventional treatment in the emergency green channel was collected retrospectively. The patients who received multimodal computed tomography (CT) were included in the CT group. Patients who underwent multimodal MRI examinations were included in the MRI group, and the door-to-needle time (DNT), neurological function, and prognosis of the two groups were compared. The result turned out that among the 126 patients included, 40 patients underwent CT examination (CT group) and 86 patients underwent MRI examination (MRI group). A comparison of general data between the CT group and the MRI group showed *P* > 0.05. The MRI group's DNT time (61.23 ± 9.32) min was shorter than that of the CT group (87.22 ± 14.26) min, *P* < 0.05. Through comparison, the *P* values of mRS scores and NIHSS scores in both groups were greater than 0.05. After treatment, the mRS score and NIHSS score of the MRI group was lower, with *P* < 0.05. According to the results of this study, it can be concluded that emergency multimodal MRI could shorten the DNT time of patients with acute and hyperacute ischemic stroke, reduce the degree of neurological impairment, and improve the prognosis.

## 1. Introduction

As the most common type of stroke, acute ischemic stroke (AIS) accounts for 69.6%–70.8% of stroke incidence in our nation [1, 2]. AIS is characterized by upper fatality rate, disability rate, and recurrence rate, which pose a great threat to patients' lives and quality of life [3]. The time of prehospital transport, posthospital examination, disease diagnosis, formulation, and implementation of treatment plans in AIS patients is closely related to the clinical efficacy and prognosis of patients. According to the American Heart and Stroke Association, the door-to-needle time (DNT) for more than 50% of ischemic stroke patients should be reduced to less than 60 minutes [4]. For AIS patients, in-hospital mortality was reduced by 5% for each 15 min reduction in DNT [5]. Rapid diagnosis of AIS can be carried out as soon as possible to implement reperfusion therapy and save the brain cells in the penumbra area as much as possible to achieve efficient treatment, which can improve the survival rate of patients. At present, stroke diagnosis and treatment centers have been established in most areas of China. Through multidepartment coordination and cooperation, the establishment of a multidisciplinary stroke diagnosis and treatment team and green treatment channel can help the efficient treatment of stroke patients. However, as many as 80% of AIS patients cannot be sent to medical institutions within 3 h of onset, resulting in most patients missing the best opportunity for thrombolysis [6]. Rapid diagnosis and treatment of stroke in China has a long way to go.

The article "Application of Multimodal Magnetic Resonance Imaging in Green Channel of Acute and Hyperacute Ischemic Stroke" was published in 2022. Journal: Contrast Media Mol Imaging.

Thrombolytic therapy for AIS is often used in clinical practice. The primary goal is timely recalculation of the responsible artery and restoration of blood perfusion to save the dying ischemic penumbra (IP) [7]. However, thrombolytic therapy has a strict time window, and reperfusion therapy cannot be performed for patients with postwake stroke who cannot determine the time of stroke, which seriously affects the prognosis and increases the disability rate and mortality rate [8]. At present, the content of the AIS clinical examination and diagnosis includes history, physical examination, imaging examination, laboratory examination, disease diagnosis, and etiological classification, etc. The imaging examination methods include emergency plain CT, multimodal CT, multimodal MRI, etc. CT examination is the preferred imaging method for ischemic stroke, but it is difficult to determine the size of the infarct core and the ischemic penumbra in patients without hemorrhage. Multimodal MRI included diffusion weighted imaging (DWI), perfusion weighted imaging (PWI), arterial spin labeling (ASL), T2 star weighted angiography (SWAN), and three-dimension time of flight MRA (3D-TOF MRA). It can accurately assess the infarction core area and IP range and has important application value in the assessment of responsible artery location, thrombosis, and onset time [9]. At present, there are few reports on the application of multimodal MRI in the AIS. Therefore, the study attempted to discuss the application of multimodal magnetic resonance technology in the green channel of acute and hyperacute ischemic stroke and provide an imaging basis for the clinical treatment and prognosis evaluation of acute and hyperacute ischemic stroke.

The article "Application of Multimodal Magnetic Resonance Imaging in Green Channel of Acute and Hyperacute Ischemic Stroke" was published in 2022. Journal: Contrast Media Mol Imaging.

## 2. Materials and Methods

### 2.1. Patients with Source

The clinical data of acute and hyperacute ischemic stroke patients who received interventional treatment in the emergency green channel in our hospital from February 2020 to October 2021 were retrospectively analyzed. This study was approved by the Medical Ethics Committee of our hospital, and all patients gave informed consent. Inclusion criteria: (1) acute or hyperacute ischemic stroke was diagnosed according to relevant clinical diagnostic criteria [10]. (2) The time between the onset of symptoms and MRI or CT examination was less than 24 hours; (3) complete baseline data and the records of DNT, neurological function, and prognosis; (4) patients had good compliance during treatment; (5) aged over 18 years old. Exclusion criteria: (1) contraindications for magnetic resonance examination; (2) abnormal function of liver and kidney and other important organs; (3) previous history of arteriovenous malformation, intracranial hemorrhage or intracranial aneurysm; (4) coma or critical condition (NIHSS >25 points) [11]; (5) the presence of mental disorders or communication disorders. A total of 126 patients were enrolled, including 61 males and 65 females. The age ranged from 45 to 76 years, with an average of 65.55 ± 6.37 years. Clinical manifestations: 70 cases of dizziness, 56 cases of hemiplegia, 45 cases of partial numbness, 37 cases of slurred speech. Previous medical history: 71 cases of hypertension, 28 cases of diabetes, 54 cases of coronary heart disease, 89 cases of abnormal lipid metabolism, and 40 cases of stroke. Preoperative systolic blood pressure was 147.26 ± 25.53 mmHg, and admission diastolic blood pressure was 85.26 ± 14.38 mmHg. All of the studies were conducted without extending patients' DNT. The detailed steps of this study were shown in Figure 1.

### 2.2. Collection of Baseline Data, DNT, Neurological Function, and Prognosis

Baseline data and records of DNT, neurological function, and prognosis were collected. (1) Baseline data included sex, age, and nature of ischemic brain death (acute/hyperacute). (2) Neurological function: three months before and three months after treatment, the National Institutes of Health Stroke Scale (NIHSS) [12] score was used to evaluate, with a total score of 0–42, which included visual field, consciousness level, facial paralysis, upper and lower limb movement, ataxia, and the score was positively proportional to the degree of neurological impairment. (3) Prognosis and outcome: 3 months before and 3 months after treatment, the Modified Rankin Scale (mRS) [13] was applied, with a total score of 6. Death was rated 6 points. Bedridden or fecal incontinence or severe disability were rated as 5 points. Unable to take care of their own body or severe disability were rated as 4 points. Without help walking or moderate disability were rated as 3 points. Mild disability or being unable to complete all previous activities were rated as 2 points. No obvious functional disability or symptoms were rated as 1 point. No symptoms as evaluated at 0. mRS score >2 was classified as poor prognosis, and mRS score ≤2 was classified as good prognosis.

The article "Application of Multimodal Magnetic Resonance Imaging in Green Channel of Acute and Hyperacute Ischemic Stroke" was published in 2022. Journal: Contrast Media Mol Imaging.

### 2.3. Inspection Methods and Image Analysis

Patients who met the inclusion criteria were examined by green channel MRI related sequence examination using a GE Discovery 750 3.0T MRI scanner with a 32-channel cranial coil. The scanning sequence included T1WI, T2WI, PWI, T2WI fluid-attenuated inversion recovery (T2Flair), DWI, SWAN, and 3D-TOF MRA. (1) Specific DWI parameters: the TR 2000 ms, TE 145 ms, the matrix 416 × 320, FOV 26, layer thickness 2 mm. (2) Specific parameters of SWAN scanning: TR 37.4 ms, TE 22.9 ms, matrix 416 × 320, layer thickness 2 mm, spacing 0 cm, collection times 1, NEX 0.70, bandwidth 62.5 KHz, and reverse angle 20°. (3) Specific parameters of 3D-TOF MRA sequence: the TR 21 ms, TE 2.5 ms, FOV 18, NEX 1, reverse Angle 15°, matrix 320 × 224. (4) For postwake stroke and stroke with unknown onset time, T2 FLAIR sequence was increased, with specific parameters: TR 8500 ms, TE 145 ms, matrix 256 × 224, FOV 26, layer thickness 5 mm, NEX 1. Check time: DWI 10 “, SWAN 2 ′43”; 3D-TOF MRA 2 ′35 “; FLAIR 1 ′51”. Total examination time 5 ′04 “, add FALRI sequence to 6′ 55”.

The original data of SWAN was processed by minimum density projection (MinIP) using Funcool 4.6 software. (1) The vascular shadow with significantly lower signal and increased torsion around the core area of high signal infarction in diffusion weighted imaging (DWI) in SWAN diagram was defined as protruding vascular sign (PVS). (2) The spot-like or strip-like low signal in the transitional area of the responsible artery was defined as magneto-sensitive vascular sign (SVS), and the spot-like or lump-like low signal in the ischemic infarction area was defined as bleeding transformation (HT). (3) The area displayed as high signal in DWI sequence and low signal in ADC image was determined as the core area of infarction.

Image processing was evaluated independently by two associate chief radiologists and reevaluated by another associate chief radiologist or chief radiologist when inconsistent results occurred.

### 2.4. Statistical Methods

The SPSS 23.0 software was applied to analyze the data. The measurement data conforming to normal distribution are represented by mean ± standard deviation, and *t*-test was applied. Cases or percent were used to represent the count data, applying the chi-square test. The inspection level was *α* = 0.05.

The article "Application of Multimodal Magnetic Resonance Imaging in Green Channel of Acute and Hyperacute Ischemic Stroke" was published in 2022. Journal: Contrast Media Mol Imaging.

## 3. Results

### 3.1. Grouping and General Data Comparison

Among the 126 patients included, 40 patients underwent CT examination (CT Group) and 86 patients underwent MRI examination (MRI Group). The general data of the two groups were compared, *P* > 0.05, indicating comparability. The general data of the two groups were shown in Table 1. The MRI image of a patient was shown in Figure 2.

### 3.2. The DNT Time of Multimodal MRI Examination Was Shortened

The DNT time of MRI group (61.23 ± 9.32) min was shorter than that of CT group (87.22 ± 14.26) min, with *P* < 0.05. Comparison of DNT time between the two groups is shown in Table 2 and Figure 3.

### 3.3. The mRS Score Decreased More Significantly in Patients Undergoing Multimodal MRI Examination

Comparison of mRS scores between the two groups before treatment, *P* > 0.05. After treatment, mRS score of MRI Group was lower, *P* < 0.05. MRS scores of MRI Group and CT Group were shown in Table 3 and Figure 4.

### 3.4. The NIHSS Scores Decreased More Significantly in Patients Undergoing Multimodal MRI Examination

Comparison of NIHSS scores between the two groups before treatment, *P* > 0.05. After treatment, NIHSS scores of MRI Group was lower, *P* < 0.05. MRS scores of MRI Group and CT Group are shown in Table 4 and Figure 5.

## 4. Discussion

Cells in the AIS infarct area would cause nerve damage due to hypoxic ischemic necrosis. However, due to the abundant blood supply and collateral circulation of brain tissue, there were still a large number of active nerve cells in the cerebral infarction area at the early stage of AIS [14]. The clinical treatment of AIS was to recalculate the responsible artery to restore blood perfusion. For example, thrombolytic therapy was given to patients within an effective time window to restore blood supply to the ischemic area, save the undead nerve cells in the infarction core area, and promote the recovery of nerve function, which was crucial to improving the prognosis of injured patients [15,16]. Rapid examination and effective treatment were the keys in AIS diagnosis and treatment. Multimode MRI could compensate for the limitations of multimode CT in the examination of infarct core size and ischemic penumbra [17]. Therefore, this study analyzed the application value of multimode MRI in the green channel of acute and hyperacute ischemic stroke.

Postwaking stroke referred to the absence of stroke symptoms before sleep and the presence of stroke symptoms after awakening [18]. Since the timing of onset could not be determined, reperfusion therapy could not be performed in these patients, making it difficult to achieve a good prognosis. Multimodal imaging assessment was the basis of individual patient selection. This study retrospectively analyzed the clinical data of patients with acute and hyperacute ischemic stroke, and compared them with multimodal CT examination to observe the effect of multimodal MRI examination. And it turns out that the DNT time of patients with multimodal MRI was shortened [(61.23 ± 9.32) min vs. (87.22 ± 14.26) min], and mRS score and NIHSS score were reduced after treatment, suggesting that multimodal MRI could shorten DNT time, reduce the degree of neurological impairment, and improve the prognosis. It was consistent with relevant research results [19,20]. Multimode MRI includes DWI, PWI, etc. (1) DWI could observe the flow and diffusion of microscopic water molecules. When the membrane function of cerebral ischemic tissue was abnormal, the Brownian motion of water molecules and cell edema was weakened. At this time, DWI imaging shows high signal intensity, indicating that the ischemic brain tissue was in the stage of cytotoxic edema. In addition, DWI could detect ischemic lesions in time within minutes of symptom onset. Therefore, DWI could determine the size, location, and onset time of lesions at the early stage of AIS, and had high sensitivity in the examination of small infarcts at the early stage of AIS, shortening the DNT time of patients [21]. (2) Positive DWI and negative T2 fluid-attenuated inversion recovery (T2 FLAIR) indicated the onset of the patients within 4.5 h. It had also been recommended as an effective indicator for judging the time window of stroke patients with unknown onset, so as to achieve individualized treatment [22]. (3) PWI could display cerebral hemodynamic status. When patients had a mismatch between diffusion and perfusion, and PWI shown a hypoperfusion area but no corresponding dispersion abnormality, the presence of ischemic penumbra may be suggested. Timely intravenous thrombolytic therapy at this time was helpful to improve the prognosis [23]. (4) AIS could be caused by various components of thrombosis, including white thrombus, red thrombus, and mixed thrombus. White thrombus was mainly composed of platelets and fibrin, while red thrombus was rich in red blood cells. Due to differences in pathological mechanism and hemodynamics, cardiogenic emboli were mainly composed of red thrombi, while arteriosclerotic thrombi were mainly composed of white thrombi [24]. Red thrombi contained a large amount of deoxyhemoglobin. As paramagnetic substances, red thrombi could lead to changes in local magnetic field, which could be shown as low signal shadows whose diameters exceeded that of the contralateral vessels in SWAN. This imaging sign was known as susceptibility vessel sign (SVS). The larger diameters of the corresponding vessels on the contralateral side were related to the “halo effect” [25]. Meanwhile, SWAN phase diagram and magnetic sensitivity quantitative diagram could help distinguish calcified and noncalcified emboli [26]. (5) When FLAIR had no obvious abnormal signal but DWI shown high signal (DWI does not match FLAIR), the time window of the patient's onset tissue could be determined, indicating that the patient's brain tissue was in the stage of ischemic edema. At this time, thrombolysis was given to the patient to make the tissue reperfusion after ischemia, so as to save part of the brain tissue and reduce the degree of neurological impairment [27]. (6) The 3D-TOF-MRA was based on the signal difference between flowing blood and stationary brain tissue [28]. With high resolution, it could clearly display large and small blood vessel blockages, and had many advantages such as noninvasive, simple operation, and fast inspection speed. It could also be observed by rotating from multiple angles to fully display intracranial large vessels and branches [29]. It could provide effective basis for clinical diagnosis and interventional therapy to evaluate whether narrow or occluded and the degree of lesion.

The article "Application of Multimodal Magnetic Resonance Imaging in Green Channel of Acute and Hyperacute Ischemic Stroke" was published in 2022. Journal: Contrast Media Mol Imaging.

## 5. Strengths and Limitations

The advantage of this study was that it explored the application of multimodal magnetic resonance technology in the green channel of acute and hyperacute ischemic stroke and obtained good results. However, there were also shortcomings, which were that the sample size was relatively small, the enrolled patients were all noncritical patients, and the examination time was within 24 hours after admission. As a consequence, the determination of PVS could not be quantified yet, and it was subjective to some extent. It is expected to be further improved in future applications.

## 6. Conclusions

In conclusion, according to the results of this study, it can be concluded that emergency multimodal MRI could shorten the DNT time of patients with acute and hyperacute ischemic stroke, reduce the degree of neurological impairment, and improve the prognosis. This paper discussed the application of multimodal MRI value, and the study had obtained a good effect, and the predecessors' research results were basically consistent. Therefore, this study was a step forward on the basis of previous research results. This study could provide new ideas and guidance for the treatment of acute and hyperacute ischemic strokes in the green channel, which has research significance.

The article "Application of Multimodal Magnetic Resonance Imaging in Green Channel of Acute and Hyperacute Ischemic Stroke" was published in 2022. Journal: Contrast Media Mol Imaging.

## Figures and Tables

**Figure 1:** The detailed steps of this study. Note: DNT = door-to-needle time, mRS = modified Rankin Scale, and NIHSS = NIH Stroke Scale.

**Figure 2:** MRI image of a patient. Note: the patient was a 49-year-old man with impaired right limb movement and slurred speech for 2 hours. In (a) and (b), DWI shows patchy higher signal intensity in the left frontal lobe, insula, and lateral ventricular asides (hyperacute ischemic stroke). In (c) and (d), ADC suggests patchy low signal in the voiceover area of the left frontal lobe, insula, and lateral ventricle. In (e)–(h), SWAN indicates increased distribution of draining and decreased signal of left frontal temporal lobe and insular pia meningeal. In addition, the distribution of medullary veins in the voiceover area of the lateral ventricle increased and signal decreased (positive PVS). In (I) and (j), 3D-TOF MRA suggests occlusion of the M1 segment of the left middle cerebral artery.

**Figure 3:** DNT time. Note: there were 40 cases in CT Group and 86 cases in MRI Group. ^*∗*^represents data comparison, *P* < 0.05.

**Figure 4:** mRS scores. Note: there were 40 cases in CT Group and 86 cases in the MRI Group. ^*∗*^represents data comparison, *P* < 0.05.

**Figure 5:** NIHSS scores. Note: there were 40 cases in CT Group and 86 cases in MRI Group. ^*∗*^represents data comparison, *P* < 0.05.

**Table 1:** Comparison of general information between the two groups.

General information	CT Group(*n* = 40)	MRI Group(*n* = 86)	t/*χ*^2^	*P*
Gender(male/female)	(25/15)	(40/46)	2.794	0.095
Age (year, $\bar{x}$ ± *s*)	65.49 ± 6.24	65.61 ± 6.50	0.098	0.922
Ischemic stroke (acute/hyperacute)	(29/11)	(62/24)	0.002	0.962
Clinical manifestation (dizziness/hemiplegia/partial numbness/slurred speech)	(22/17/14/15)	(48/39/31/22)	1.276	0.735
Previous medical history (hypertension/diabetes/coronary heart disease/abnormal lipid metabolism/stroke)	(23/9/17/28/17)	(48/19/37/61/23)	1.782	0.776
Preoperative systolic blood pressure (mmHg, $\bar{x}$ ± *s*)	146.51 ± 30.06	148.01 ± 21.00	0.324	0.509
Admission diastolic blood pressure (mmHg, $\bar{x}$ ± *s*)	86.06 ± 10.17	84.46 ± 18.59	0.747	0.611

**Table 2:** Comparison of DNT time between the two groups (min,‾*x* ± *s*).

Group	Number of cases	DNT time
CT group	40	87.22 ± 14.26
MRI group	86	61.23 ± 9.32
*t*		12.220
*P*		＜0.001

**Table 3:** Comparison of mRS scores between the two groups (point, ‾*x* ± *s*).

Group	Number of cases	mRS scores	
		Before treatment	After treatment
CT group	40	2.95 ± 0.61	1.50 ± 0.28
MRI group	86	2.98 ± 0.55	1.28 ± 0.32
*t*		0.275	3.732
*P*		0.784	＜0.001

**Table 4:** Comparison of NIHSS scores between the two groups (point, ‾*x* ± *s*).

Group	Number of cases	NIHSS scores	
		Before treatment	After treatment
CT group	40	8.91 ± 1.53	3.65 ± 0.47
MRI group	86	8.90 ± 1.55	2.96 ± 0.58
*t*		0.034	6.582
*P*		0.973	＜0.001

The article "Application of Multimodal Magnetic Resonance Imaging in Green Channel of Acute and Hyperacute Ischemic Stroke" was published in 2022. Journal: Contrast Media Mol Imaging.

## Data Availability

The data used to support the findings of this study are available from the corresponding author upon request.
